The article "miR-126a-3p induces proliferation, migration and invasion of trophoblast cells in pre-eclampsia-like rats by inhibiting A Disintegrin and Metalloprotease 9" was retracted in 2020. Reason: duplicated images.

# miR-126a-3p induces proliferation, migration and invasion of trophoblast cells in pre-eclampsia-like rats by inhibiting A Disintegrin and Metalloprotease 9

**DOI:** 10.1042/BSR20191271

**Published:** 2019-12-20

**Authors:** Shenglong Zhao, Jiandong Wang, Zheng Cao, Lei Gao, Yuanyuan Zheng, Jing Wang, Xiaowei Liu

**Affiliations:** 1 Obstetrics Department, Beijing Obstetrics and Gynecology Hospital, Capital Medical University, Beijing 100026, P.R. China; 2 Gynecologic Oncology Department, Beijing Obstetrics and Gynecology Hospital, Capital Medical University, Beijing 100026, P.R. China; 3 Clinical Laboratory, Beijing Obstetrics and Gynecology Hospital, Capital Medical University, Beijing 100026, P.R. China

**Keywords:** ADAM9, biological characteristics, miR-126a-3p, preeclampsia, trophoblast cells

## Abstract

The present study aimed to investigate the underlying mechanism of miR-126a-3p in the proliferation, migration and invasion of trophoblast cells in pre-eclampsia-like rats by targeting A Disintegrin and Metalloprotease 9 (ADAM9). First, the interaction between miR-126a-3p and ADAM9 was confirmed via biochemical assays. Placental tissues and trophoblast cells were then obtained. RNA *in situ* hybridization was performed in order to detect miR-126a-3p expression in the placenta. Subsequently, a series of biological assays, including reverse transcription-quantitative PCR (RT-qPCR), Western blotting, MTT assay, apoptosis assay, cell cycle assay, wound healing assay and transwell assay were adopted in order to determine the cell proliferation, cell cycle distribution, apoptotic rate, and migration and invasion of trophoblast cells in each group. The results revealed that miR-126a-3p was down-regulated in the placenta of pre-eclampsia-like rats. *In vivo* experiments’ results indicated that miR-126a-3p could inhibit ADAM9 expression, and induce cyclin D1, Matrix metalloproteinase (MMP) 2 (MMP-2), MMP-9 expression. MTT, apoptosis and cell cycle assay results revealed that trophoblast cells transfected with miR-126a-3p mimic or si-ADAM9 exhibited higher proliferative activity and a lower apoptotic rate compared with the blank group (all *P*<0.05). The wound healing assay and transwell assay results confirmed that, compared with the blank group, the migration and invasion ability of trophoblast cells in the miR-126a-3p mimic group and small interfering RNA (siRNA)-ADAM9 group were significantly increased (all *P*<0.05). Conversely, miR-126a-3p inhibitor treatment revealed the opposite effect (all *P*<0.05). In conclusion, the present study demonstrated that miR-126a-3p could enhance proliferation, migration and invasion, but decrease the apoptosis rate of trophoblast cells in pre-eclampsia-like rats through targeting ADAM9.

The article "miR-126a-3p induces proliferation, migration and invasion of trophoblast cells in pre-eclampsia-like rats by inhibiting A Disintegrin and Metalloprotease 9" was retracted in 2020. Reason: duplicated images.

## Introduction

Pre-eclampsia, as a high blood pressure disease, is characterized by new-onset of hypertension, proteinuria, headache, vomiting and nausea after 20 weeks of gestation [1]. When the disease gets more serious, individuals suffer from pre-eclampsia frequently, accompanied by multiple organ disorders [2]. Furthermore, pre-eclampsia is regarded as an important cause of fetal and maternal deaths, but currently, there are no effective methods available for treating pre-eclampsia, other than premature termination of pregnancy or delivery [3,4]. Accumulating evidence indicates that pre-eclampsia is primarily associated with the uterine spiral artery remodeling disorder caused by insufficient infiltration of trophoblast cells [5]. As the most important cell type in the placental tissue, any biological abnormalities in trophoblast cells would easily lead to developmental defects in the placenta [6]. Peng et al. [7] reported that pre-eclampsia is often accompanied by excessive apoptosis of trophoblast cells, which is positively correlated with the severity of maternal disease. Therefore, in order to establish a novel therapeutic strategy for pre-eclampsia, it is essential to investigate the molecular mechanisms underlying the formation and progression of pre-eclampsia.

microRNAs are endogenous, small, non-coding RNA sequences that have a number of regulatory functions in human cells [8]. It has been verified that miRNAs may serve a prominent role in the progression of placental growth and functional regulation [9]. miR-126 is a common angiogenesis-associated RNA in humans. Yan et al. [10] demonstrated that miR-126 could promote the growth of vascular endothelial cells and placental blood vessels in pre-eclampsia. Another study demonstrated that miR-126-3p plays an important role in the regulation of placental angiogenesis in pre-eclampsia [11]. However, the impact of miR-126 in pre-eclampsia remains largely unknown and warrants further investigation.

A Disintegrin And Metalloprotease 9 (ADAM9), a member of the type 1 trans-membrane protein, has been observed with significantly increased expression in various different types of tumor, such as liver cancer, breast cancer and prostate cancer [12–14]. Pre-eclampsia is a common disease leading to kidney damage, and a previous study revealed that ADAM9 affects the physiological morphology of renal tubular epithelial cells, suggesting its potential value in regulating kidney damage [15]. Another previous study demonstrated that ADAM9 exhibits abnormal expression in pre-eclampsia, as the probability of mutations in the ADAM9 gene in pre-eclampsia was approximately three times higher than that of normal puerperae [16], indicating that ADAM9 may be involved in the regulation of pre-eclampsia.

The article "miR-126a-3p induces proliferation, migration and invasion of trophoblast cells in pre-eclampsia-like rats by inhibiting A Disintegrin and Metalloprotease 9" was retracted in 2020. Reason: duplicated images.

Regardless of the discovery of a number of pre-eclampsia-associated miRNAs in recent years, there is inadequate information on their detailed cellular functions and mechanisms of action. Thus, in the present study, it was proposed that miR-126a-3p may be a prominent modulator for pre-eclampsia, potentially through interactions with its target gene, with the aim of identifying a new potential target for pre-eclampsia treatment.

## Materials and methods

### Bioinformatics prediction of molecular mechanism in pre-eclampsia

The gene expression chips were searched for in the sub database Gene Expression Omnibus (GEO; http://www.ncbi.nlm.nih.gov/geo) using the key word ‘preeclampsia’. Among the various associated chips, GSE84260 (https://www.ncbi.nlm.nih.gov/) was selected for screening differentially expressed genes. The chip contains the miRNA expression data of 32 placental tissues from pregnant women (16 pre-eclamptic women and 16 normotensive women). The datasets were processed with background correction and normalization using the Robust multiarray average (RMA) and Affy package (http://www.bioconductor.org/packages/release/bioc/html/affy.html) [17]. Subsequently, R limma package (http://master.bioconductor.org/packages/release/bioc/html/limma.html) was used to identify differentially expressed miRNAs in pre-eclampsia, and the adjusted *P*-value (p.adj) for false discovery rate correction was set as 0.01 and the log2 fold change (log2FC) absolute value was set as 2 in order to analyze the significantly differentially expressed miRNAs, and these were presented in a heat map. The three miRNA–mRNA association prediction tools, miRWalk (http://mirwalk.umm.uni-heidelberg.de/), miRSearch (https://www.exiqon.com/miRSearch) and TargetScan (http://www.targetscan.org/vert_71/), were utilized to predict the miRNA–mRNA interaction and the regulation of miRNAs to their target genes in pre-eclampsia. Venny 2.1 (http://bioinfogp.cnb.csic.es/tools/venny/index.html) was applied to draw Venn diagrams for overlapping genes from three tools [18].

### Target gene prediction and verification

Binding sites between the target gene and miR-126a-3p were displayed using the online miRNA prediction tool TargetScan (http://www.targetscan.org). ADAM9 was identified as a potential miR-126a-3p direct target gene linked to pre-eclampsia, and luciferase reporting system was applied for experimental validation. The synthetic wild-type (WT) ADAM9-3′ untranslated region (3′UTR) or mutant (MUT) ADAM9-3′UTR gene fragments with two enzyme sites, XhoI and BamHI, were amplified and inserted into the pGL4.13 report vector using restriction endonucleases and T4 DNA ligase (E6681; Promega Corp.). HEK-293T cells (BNCC338274; American Type Culture Collection) were cultured in 96-well plates, and when the confluence reached 80–90%, cells were co-transfected with the pGL4.13 report vector containing WT-ADAM9-3′UTR (MUT-ADAM9-3′UTR) and miR-126a-3p mimic (scrambled negative control). At 48 h post-transfection, cells were added using the Luc-Pair™ Firefly Luciferase HS Assay kit (LF008; iGeneBio) and fluorescence intensity was measured using GloMax®-20/20 Luminometer detector (E5311; Promega Corp.).

The article "miR-126a-3p induces proliferation, migration and invasion of trophoblast cells in pre-eclampsia-like rats by inhibiting A Disintegrin and Metalloprotease 9" was retracted in 2020. Reason: duplicated images.

### RNA pull-down

In line with the Magnetic RNA-Protein Pull-Down kit (Pierce; Thermo Fisher Scientific, Inc.), 1 μg biotin-labeled RNA was added in an Eppendorf (EP) tube along with 500 μl structure buffer. The tube was bathed in water at 9°C for 2 min and then in ice for 3 min. A total of 50 μl suspension containing magnetic beads was added in an EP tube to suspend the magnetic beads at 4°C overnight, and then the mixture was centrifuged at 3000 rpm for 3 min at 4°C. The supernatant was discarded. It was then rinsed in 500 μl washing buffer three times, added to 10 μl cell lysate, and stored at room temperature for 1 h. The incubated magnetic bead–RNA–protein mixture was centrifuged at low speed at 4°C, and the supernatant was collected and rinsed three times with 500 μl washing buffer for 5 min each time. A total of 10 μl cell lysate supernatant was taken as input. The protein concentration was measured according to the protocol from the Pierce™ BCA Protein Assay kit (23227; Thermo Fisher Scientific, Inc.). After that, protein expression was detected using Western blotting. Rabbit anti-Argonaute 2 (Ago2) (2 μg/ml; catalog no. ab32381; Abcam) and goat anti-rabbit IgG (1:2000; catalog no. ab205718; Abcam) were used as antibodies.

### Animal model construction

A total of 60 specific-pathogen free (SPF) SD rats (male:female ratio, 1:2) weighing between 200 and 220 g were obtained from the Guangdong Experimental Animal Center for use in the present study. Rats were housed in the following conditions: 12-h light and dark cycle; temperature, 18–26°C; relative humidity, 40–70%; noise, <85 db; and ammonia concentration, <20 ppm. Ventilation was changed 8–12 times/h. All rats underwent a week’s period of feeding prior to the commencement of experimentation. Each cage was housed with female and male rats at a ratio of 2:1 and the vaginal smear was performed on the following morning. The day when sperm was observed was defined as the day 0 of gestation. The 40 female rats were randomly divided into l-NAME group (30 rats) and control group (10 rats) on the 8th day of gestation. Rats in the l-NAME group received daily subcutaneous injections of l-nitro-arginine methylester (D0819; Sigma–Aldrich; Merck KGaA) 100 mg/(kg.day) once a day starting from the 10th day. Rats in the control group were injected with the same amount of normal saline at the same time point. After the 18th day, High-Field Dynamic Contrast-Enhanced MRI was performed for rats in two groups in the light of protocols [19–22]. After the physiological indexes were measured, pentobarbital sodium with high concentration (250 mg/kg) was injected into the abdomen of rats. If there was no cardiac arrest, no spontaneous breath continuing 2–3 min and no blinking reflex in rats, euthanasia was successfully carried out.

The article "miR-126a-3p induces proliferation, migration and invasion of trophoblast cells in pre-eclampsia-like rats by inhibiting A Disintegrin and Metalloprotease 9" was retracted in 2020. Reason: duplicated images.

### Blood pressure measurement

A rat tail blood pressure measuring instrument (CODE) was utilized to detect the blood pressure of the two groups at baseline and after l-NAME injection (on the 6th and 18th days of gestation). The measurements were performed as follows: the rats were deprived of water and food for 2 h prior to blood pressure measurement, which was performed at 8:00 a.m. With the incubator preheated to 37°C, the rats were placed in an incubator to adapt for 10 min. During the blood pressure measurement, the temperature of the incubator was guaranteed to be ∼25°C. The measurement was repeated three times independently.

### Urine protein detection

Urine was collected from each group at baseline and after l-NAME injection (on the 6th and 18th days of gestation) and detected using a total protein assay kit (SNM153; Biolab). The procedure was as follows: the standard curve was drawn, 18 blank tubes were divided into three groups on average and protein standard was added into each tube with a volume gradient (0.0, 0.2, 0.4, 0.6, 0.8 and 1.0 ml). ddH_2_O was supplemented into tubes until the total volume reached 1 ml, and then 4 ml Biuret was added. The mixture was incubated for 30 min at room temperature, and the optical density value at 540 nm was measured using a SpectraMax iD3 multi-function microplate reader (Molecular Devices). The first tube without the protein solution was used as the negative control. The average of the results for the three groups was taken, and a standard curve was drawn. The urine was centrifuged for 2000 rpm at 4°C for 10 min, and the supernatant was removed. The subsequent detection method was the same as that aforementioned. The experiment was repeated in triplicate.

### Isolation, culture and transfection of placental trophoblast cells

Placental tissues were taken from each group on the 21st day of gestation and made into 3 mm × 3 mm tissue sections. The sections were rinsed with D-Hank’s solution at 4°C, and DMEM low-glucose medium was added containing 0.15% collagenase with the supernatant discarded. Tissue sections were then transferred to sterile centrifuge tubes, digested for 30 min using a 37°C thermostatic electromagnetic stirrer and centrifuged at 1200 rpm at 4°C for 5 min. DMEM low-glucose medium containing 20% fetal bovine serum was added to the sections after the supernatant was removed, and centrifuged at 1200 rpm at 4°C for 5 min. A cell suspension was made by adding the precipitate to the medium. The suspension was transferred to a disposable culture dish after mixing, rinsed with D-Hank’s solution, 0.25% trypsin (containing 0.02% EDTA) added, and kept in a 5% CO_2_ and 95% air incubator at 37°C for 7–9 min. The digestion was suspended by adding DMEM containing 20% fetal bovine serum and the suspension was centrifuged at 1200 rpm for 5 min at room temperature. The supernatant was discarded and the cells were resuspended in DMEM containing 20% fetal bovine serum. The cells were then seeded into a new culture dish and incubated at 37°C, 5% CO_2_ and 95% air. The culture medium was replaced every 3 days [23].

The article "miR-126a-3p induces proliferation, migration and invasion of trophoblast cells in pre-eclampsia-like rats by inhibiting A Disintegrin and Metalloprotease 9" was retracted in 2020. Reason: duplicated images.

### Identification of placental trophoblast cells

Trophoblast cells were seeded into sterile slices (22 mm × 26 mm) and placed in a 24-well culture plate. The slices were cultured for 48 h, and washed with PBS three times, 5 min per time. The cells were then fixed with paraformaldehyde for 15 min at room temperature and rinsed with PBS three times, 5 min per time, subsequently cleared with PBS containing 0.2% Triton X-100 three times, 5 min per time. The plate then had 1% rabbit serum added to it and was sealed at room temperature for 30 min. After PBS washing, rabbit anti-mouse cytokeratin 7 (1:8000; catalog no. ab181598; Abcam) and vimentin (1:100; catalog no. ab92547; Abcam) were also added, and the plate was incubated in a shaking bed overnight at 4°C. The slices were rinsed with PBS three times, 5 min per time and incubated with Alexa Fluor® 488–conjugated goat anti-rabbit IgG (1:200; catalog no. ab150077; Abcam) as the secondary antibody in a shaking bed at 4°C for 2 h. After diluting with DAPI solution (1:1000), the slices were incubated for 1 h at room temperature. Finally, the slices were rinsed with PBS three times, 5 min per time and observed in an inversion fluorescence microscope (IX71; Olympus) to detect fluorescence and capture images. Image-Pro Plus software (version 7.0; Media Cybernetics), a software for imaging analyses, was adopted in order to determine the percentage of green fluorescent cells.

### RNA *in situ* hybridization

HRP-labeled complementary strand probes with miR-126a-3p were customized by Thermo Fisher Scientific, Inc. The placental tissue was fixed at room temperature for 24 h with 4% formaldehyde containing a neutral buffer and subsequently paraffin embedded and sectioned. Preheated probes at 55°C were added to the hybrid buffer, which was then preheated for 15 min and diluted with formamide ion removal. The slices were placed in a wet box containing buffer and hybridized for 2 h at 55°C. The sections were then washed with 1× ssc-0.1% (V/V) SDS twice for 5 min, followed by washing a further two times with 0.2× ssc-0.1% (V/V) SDS wash. After that, the sections were washed for 5 min in the detection buffer, 50 μl DAB chromogen was added to the detection buffer, and then DAPI staining was performed for staining of the nuclei. The sections were then sealed and stained under an optical microscope. The scoring criteria for slices were as follows: The intensity of the dye color was graded as 0 (no color), 1 (light yellow), 2 (light brown) or 3 (brown), and the number of positive cells was graded as 0 (<5%), 1 (5–25%), 2 (25–50%), 3 (51–75%), or 4 (>75%). The two grades were added together and specimens were assigned to one of four levels: 0–1 score (−), 2 scores (+), 3–4 scores (++), more than 5 scores (+++). The positive expression rate was expressed as the percent of the addition of (++) and (+++) to the total number.

The article "miR-126a-3p induces proliferation, migration and invasion of trophoblast cells in pre-eclampsia-like rats by inhibiting A Disintegrin and Metalloprotease 9" was retracted in 2020. Reason: duplicated images.

### Grouping and transfection of placental trophoblast cells

Placental trophoblast cells extracted from normal rats were considered as the normal control group. Placental trophoblast cells from the l-NAME group were independently assigned into six subgroups: Blank group (no sequence transfected, *n*=5), Negative Control group (transfected with negative control sequence, *n*=5); miR-126a-3p mimic group, transfected with miR-126a-3p mimic sequence, *n*=5; miR-126a-3p inhibitor group (transfected with miR-126a-3p inhibitor sequence, *n*=5); small interfering RNA (siRNA)-ADAM9 group (transfected with siRNA-ADAM9 sequence, *n*=5); miR-126a-3p mimic+siRNA-ADAM9 group (transfected with miR-126a-3p mimic+siRNA-ADAM9 sequence, *n*=5). Prior to transfection, placental trophoblast cells (2 × 10^4^ cells) confirmed to be at the logarithmic growth phase (cells were passaged within 24–48 h) were seeded into 96-well plates. After cell confluence had reached 30–50%, they were transfected using Lipofectamine 2000 (11668027; Thermo Fisher Scientific, Inc.): 100 pmol miR-126a-3p mimic and 5 μl Lipofectamine 2000 were diluted with 250 μl serum-free medium Opti-MEM (Gibco; Thermo Fisher Scientific, Inc.) and the final concentration of miR-126a-3p mimic was 50 nmol. The mixture was added into wells and incubated at room temperature for 20 min. The plate was then preserved at 37°C with 5% CO_2_ and 95% air. After 6–8 h, a complete medium was acquired for the sake of culturing the cells for an additional 48 h before subsequent experiments were performed. The transfection sequences applied to the present study were designed and synthesized by Shanghai Jima Pharmaceutical Co., Ltd. Transfection for miR-126a-3p inhibitor and ADAM9 siRNA used the same aforementioned methods.

The article "miR-126a-3p induces proliferation, migration and invasion of trophoblast cells in pre-eclampsia-like rats by inhibiting A Disintegrin and Metalloprotease 9" was retracted in 2020. Reason: duplicated images.

### Reverse transcription-quantitative PCR

For 48 h after transfection, the trophoblast cells in each group were treated with lysis buffer (Beijing Ovia Bio) and placed on ice for lysis. Total RNA of trophoblast cells in each group was extracted with TRIzol reagent (11736-051; Invitrogen; Thermo Fisher Scientific, Inc.) according to the manufacturer’s protocol. Subsequently, the total RNA was dissolved in ultrapure water treated with diethylpyrocarbonate (E174-5G; Shanghai Haoran Biotechnology Co., Ltd.) and the optical density at 260 and 280 nm was measured using ND-1000 UV/Vis spectrophotometer (Evolution 201; Thermo Fisher Scientific, Inc.) in order to determine the quality of RNA. The GoScript™ Sensiscript RT kit (A5004; Promega Corp.) was used to reversely transcribe the RNA into cDNA. According to the manufacturer’s instructions, the RT conditions were performed as follows: 70°C for 5 min, ice bath for 2 min, 42°C for 5 min, 70°C for 8 min, frozen at −80°C; and kept for further experiments. The primers in the reverse transcription-quantitative PCR (RT-qPCR) were designed and synthesized by the Takara Biotechnology Ltd., using Premier 5.0 software. The primer sequences are presented in Table 1. The reaction was performed using a RT-qPCR platform (Bio-Rad iQ5; Bio-Rad Biotechnology) with GAPDH and U6 regarded as internal references. The reaction conditions were as follows: pre-denaturation at 95°C for 30 s, denaturation 95°C for 10 s, annealing at 60°C for 20 s and extension at 70°C for 10 s. In total, 40 cycles were performed with this RT-qPCR reaction. The expression of the relative mRNA expression of the target gene in cells were measured using the −2^ΔΔ*C*_q_^ method [24]. Each experiment was repeated in triplicate.

**Table 1:** Primer sequences used in real time-PCR

Gene	Primer sequence (5′–3′)
*miR-126a-3p*	F: 5′–TCGTACCGTGAGTAATAATGCG–3′
	R: 5′–TTAGCATGGCACTCATTATTAC–3′
*ADAM9*	F: 5′–CATCCCCCTGGTTGCGGCTG–3′
	R: 5′–TGCACGGGTGGTGGTGTGGA–3′
*cyclin D1*	F: 5′–GTTCTCGGCCAGCACCAT–3′
	R: 5′–CAGCATACAATCTCGCACC–3′
*MMP-2*	F: 5′–ATGGAGGCACGATTGGTCTG–3′
	R: 5′– GCAAAGGCATCATCCACTGTC–3′
*MMP-9*	F: 5′–GGAGATTAGGAACCGCTTGCA–3′
	R: 5′–TGAACAGCAGCACCTTACCTT–3′
*U6*	F: 5′–GTGCTCGCTTCGGCAGCACATATAC–3′
	R: 5′–AAAAATATGGAACGCTTCACGAATTTG–3′
*GAPDH*	F: 5′–GGCACAGTCAAGGCTGAGAATG–3′
	R: 5′–ATGGTGGTGAAGACGCCAGTA–3′

Abbreviation: MMP, matrix metalloproteinase.

The article "miR-126a-3p induces proliferation, migration and invasion of trophoblast cells in pre-eclampsia-like rats by inhibiting A Disintegrin and Metalloprotease 9" was retracted in 2020. Reason: duplicated images.

### Western blotting

Lysate (7 mol/l urea, 2 mol/l thiourea, 5 ml/l IPG buffer (pH 3–10), 65 mmol/l Dithiothreitol, 40 g/CHAPS, 5 mg/l protease inhibitor and 10 ml/l trypsin inhibitor) was added to the trophoblast cells. The mixture was then shaken and placed on ice for ultrasonic pulverization, centrifuged at 4°C at 12000 rpm for 30 min and the liquid supernatant taken accordingly. The protein concentration in the supernatant was determined using a BCA kit (P0009; Shanghai Biyuntian Biotechnology Co., Ltd.). The 5× SDS lysate (P0013G; Shanghai Biyuntian Biotechnology Co., Ltd.) was added and the protein was inactivated by heating for 5 min at 100°C. A total of 20 µg cell lysates were electrophoresed in a polyacrylamide gel (5% concentrated gel and 12% separating gel) and separated via SDS/PAGE (10% gel) and transferred on to NC membrane (EMD Millipore). After blocking in TBST solution containing 5% bovine serum albumin for 1 h at room temperature, membranes were then incubated with specific primary antibodies including rabbit antibody ADAM9 (1:1000; catalog no. ab186833; Abcam), cyclin D1 (1:10000; catalog no. ab134175; Abcam), Matrix metalloproteinase (MMP) 2 (MMP-2) (1 μg/ml; catalog no. ab37150; Abcam), MMP-9 (1:1000; catalog no. ab38898; Abcam) for 2 h at room temperature, and GAPDH was used as an internal reference (1:1000; catalog no. ab8245; Abcam). The membrane was then washed three times with PBS, and after incubation overnight (10 min/time), diluted secondary goat anti-rabbit antibody IgG (1:2000; catalog no. ab6721; Abcam) was added, and subsequently the membrane was incubated at 4°C for 4–6 h and washed three times with TBST buffer (15 min/time). Later, the membrane was immersed in an electro-chemi-luminescence (ECL) developing solution (32106; Thermo Fisher Scientific, Inc.) at room temperature for 1 min. Image-Pro Plus software (version 7.0) was used for the analysis of gray value for proteins. The relative protein level was evaluated by the gray value of the target protein/the gray value of GAPDH. The experiment was repeated in triplicate.

### MTT assay

Cells in the logarithmic growth phase were seeded into 96-well plates with a cell density adjusted to 1 × 10^5^ cells/ml (100 μl per well), cells were then incubated in a 5% CO_2_ and 95% air cell culture incubator at 37°C. Next, the culture plates were taken out and 10 μl of 5 mg/ml MTT solution (SBJ-0190, Nanjing Senbega Biotechnology Co., Ltd.) was added at 24, 48 and 72 h and incubated for 4 h under dark conditions. The optical density (OD) value of each well was measured at a wavelength of 570 nm with a full wavelength microplate reader (51119200; Thermo Fisher Scientific, Inc.). The experiment was repeated in triplicate.

The article "miR-126a-3p induces proliferation, migration and invasion of trophoblast cells in pre-eclampsia-like rats by inhibiting A Disintegrin and Metalloprotease 9" was retracted in 2020. Reason: duplicated images.

### Cell cycle and apoptosis detection

The culture medium was abandoned after transfection for 48 h, and cells were then washed with PBS and digested with 0.25% trypsin, cells were adjusted to 2 × 10^5^ cells/ml concentration with medium, 1 ml cell was collected and washed with PBS three times, then cells were centrifuged at 1000 rpm at 4°C for 5 min with the supernatant removed. Subsequently the cells were added to precooled anhydrous ethanol (absolute ethanol:PBS ratio, 3:1), fixed at 4°C overnight, and then washed with PBS twice and centrifuged at 1000 rpm for 5 min followed by removal of the supernatant. Cells were then added to 10 μl RNase and incubated at 37°C for 5 min. Next, 400 μl PI (P8080; Beijing Solarbio Science & Technology Co., Ltd.) was added for staining in the dark for 30 min. Subsequently the samples were placed into CytoFLEX (Cube6; Partec) to detect the period of cell proliferation at 488 nm. The experiment was repeated in triplicate.

Cell apoptosis was detected by Annexin-V-FITC/PI. After 48 h transfection, cells were adjusted to a concentration of 2 × 10^5^ cells/ml, and the cells were treated with 0.3% trypsin (without EDTA) and collected. Cells were then resuspended with 1 ml binding buffur, centrifuged at 1000 rpm at 4°C for 5 min and the supernatant removed. The Annexin-V-FITC/PI kit (CA1020-50T; Beijing Solarbio Science & Technology Co. Ltd.) was utilized to detect cell apoptosis. Each tube had 100 μl cells (total 1 × 10^5^ cells) and 5 μl Annexin-V-FITC added, and were then mixed and incubated at room temperature for 10 min. Subsequently, 5 μl PI was added and the cells were incubated again at room temperature for 5 min, and PBS was then added until the solution reached 500 μl. Apoptosis was immediately analyzed by CytoFLEX at 488 nm. The apoptosis rate was analyzed and calculated using CellQuest 3.0 (BD Biosciences). The experiment was repeated in triplicate.

### Wound healing assay

Placental trophoblast cells were collected and seeded into a 96-well plate at a density of 1 × 10^6^ after 48 h of transfection. Subsequently, the cells were cultured in a 5% CO_2_ incubator at 37°C. After the cell confluence reached ∼95%, a straight line was drawn on the 96-well plate surface under the guidance of the straight edge of a sterile gun. The cells were then rinsed with D-Hank’s solution and again cultured with serum-free medium after removing the falling cells. Samples were collected at 0 and 24 h and images were captured under an inverted microscope (IX53; Olympus) with the scratch distance measured at both 0 and 24 h after culture. The healing rate represents the cell migration ability. Healing rate (%) was calculated under the formula: (0 h scratch width − 24 h scratch width)/0 h scratch width × 100%. The experiment was repeated in triplicate.

The article "miR-126a-3p induces proliferation, migration and invasion of trophoblast cells in pre-eclampsia-like rats by inhibiting A Disintegrin and Metalloprotease 9" was retracted in 2020. Reason: duplicated images.

### Transwell assay

ECM gel (E0282; Sigma–Aldrich; Merck KGaA) was diluted with serum-free DMEM at a ratio of 1:7 and then kept in a 37°C incubator for 15 min. The cells were rinsed twice with PBS, digested with 0.25% trypsin and suspended with serum. Subsequently the cell concentration was adjusted to 2.5 × 10^4^ cells/ml using serum-free DMEM. A total of 200 μl DMEM containing 10% serum was dispensed to the Transwell lower chamber, and the upper chamber had a cell suspension at a density of 1 × 10^4^ cells/ml, and 200 μl of DMEM added. The Transwell chambers were collected after 48 h of incubation in accordance with the Transwell protocol. The polycarbonate membrane was cut out, and the bottom of the membrane was fixed with acetone at 4°C for 5 min and stained in 0.1% Crystal Violet for 20 min. The total number of cells crossing the membrane was observed under a microscope, images of each membrane were captured from five representative views and then counted. Invasion rate was calculated as the number of stained cells/total number of cells × 100%. The experiment was independently repeated three times.

### Statistical analysis

Data were analyzed using SPSS software (version 21.0; IBM Corporation). Data are presented as the mean ± standard error. Comparisons between two groups were performed using Student’s *t* test. Comparisons among multiple groups were analyzed using one-way analysis of variance. Tukey’s test was used for the post hoc multiple comparisons. Cell proliferation at different time points were compared using repeated-measures analysis of variance. *P*<0.05 was considered to indicate a statistically significant difference.

## Results

### Bioinformatics prediction of pre-eclampsia-associated miRNA and target genes

Bioinformatics tools were used in order to identify the pre-eclampsia-specific miRNAs. According to information screened from the analysis of the chip data (GSE84260), a total of 499 differentially expressed miRNAs in patients with pre-eclampsia compared with controls were identified, using |logFC| 2.0 and adj.P.Val <0.01 as the cut-off point, and the top ten most relevant differentially expressed miRNAs were selected and illustrated in the heat map (Figure 1A). Studies have revealed that miR-126 could promote pre-eclamptic placental vascular endothelial cell production and blood perfusion [10,25]. By searching the miRbase database (http://www.mirbase.org/), miR-126 in rats was named as miR-126a, which is highly homologous to miR-126. The present study selected miR-126a-3p for investigation. In order to elucidate the candidate gene targeted by miR-126a-3p, miRWalk, miRSearch and TargetScan databases were investigated, and 3717, 56 and 52 genes were identified, respectively. Data obtained from the three miRNA prediction software were presented on Venn image (Figure 1B). It was established that *PLXNB2, ADAM9, KANK2, PLK2, CRK, CAMSAP1* and *PTPN9* were intersection genes. ADAM9 mediates the physiological morphology of renal tubular epithelial cells, which may be involved in the regulation of kidney damage [15]. There are also studies demonstrating that ADAM9 is highly expressed in the anoxic environment caused by pre-eclampsia compared with normal parturients [16]. The predicted binding site of miR-126a-3p and ADAM9 is presented in Figure 1C. Data obtained from the bioinformatics analysis indicated that miR-126a-3p may influence the occurrence and development of pre-eclampsia through targeting ADAM9.

The article "miR-126a-3p induces proliferation, migration and invasion of trophoblast cells in pre-eclampsia-like rats by inhibiting A Disintegrin and Metalloprotease 9" was retracted in 2020. Reason: duplicated images.

**Figure 1:** Screening of key pre-eclampsia-associated miRNAs and genes via bioinformatics analysis (**A**) Venn diagrams presenting the top ten differentially expressed miRNAs. The x-axis indicates the sample number, the y-axis presents the differentially expressed miRNAs. The key for the color scheme is present at the right panel with each rectangle corresponding to an individual sample. The red and blue colors indicate relatively high and low fold-change of expression, respectively. (**B**) miRWalk, miRSearch and TargetScan were used to identify pre-eclampsia-associated genes targeted by miR-126a-3p; PLXNB2, ADAM9, KANK2, PLK2, CRK, CAMSAP1 and PTPN9 were selected. (**C**) TargetScan predicts ADAM9 as an miR-126a-3p target gene.

### miR-126a-3p down-regulates ADAM9 expression

The target association between miR-126a-3p and ADAM9 was further verified via a Luciferase assay (Figure 2A). As indicated in Figure 2A, a significant decrease in luciferase activity was observed in HEK-293 cells co-transfected with luciferase reporter vector containing miR-126a-3p mimic and ADAM9 3′UTR-WT plasmid compared with cells transfected with negative control and ADAM9-3′UTR-WT sequence (*P*<0.05). No significant difference was observed among the other groups (all *P*>0.05). Such results provided direct evidence that miR-126a-3p negatively regulates ADAM9 expression.

**Figure 2:** Verification of miR-126a-3p target site on ADAM9 (**A**) The binding sites of miR-126a-3p and ADAM9 were verified using a luciferase reporter gene assay. HEK-293T cells were cultured in 96-well plates and then co-transfected with luciferase reporter WT or MUT plasmid, as well as NC or miR-126a-3p mimic sequence when cell confluence reached 80–90%. The luciferase activity was detected 48 h after transfection. (**B**) Verification of ADAM9 binding to Ago2 by RNA pull-down. Total protein was extracted from HEK-293T after cell lysis, followed by an RNA pull-down test according to the protocol of the kit. (**C**) Relative expression of proteins for RNA pull-down. (**D**) Total RNA was extracted from trophoblast cells 48 h after transfection, and the relative mRNA expression of miR-126a-3p and ADAM9 were determined via RT-qPCR analysis. (**E**) Bands of ADAM9 protein. (**F**) The total protein level of trophoblast cells in each group was extracted after 48 h transfection, and the relative protein expression of ADAM9 was determined via Western blotting. *P<0.05 vs. NC and ADAM9-3′UTR group; ^#^*P*<0.05 vs. negative control group. The experiments were repeated in triplicate.

The article "miR-126a-3p induces proliferation, migration and invasion of trophoblast cells in pre-eclampsia-like rats by inhibiting A Disintegrin and Metalloprotease 9" was retracted in 2020. Reason: duplicated images.

Ago2 can promote the process of the RNA-induced silencing complex (RISC) and mediates siRNA-directed mRNA cleavage and miRNA translational suppression. RNA pull-down analysis was utilized to confirm the potential binding of ADAM9 and Ago2; as indicated in Figure 2B,C, Ago2 directly interacts with ADAM9.

In order to further confirm the suppression of ADAM9 by miR-126a-3p *in vitro*, RT-qPCR and Western blotting were performed and the results revealed that, compared with the negative control group, the miR-126a-3p mimic group demonstrated significantly decreased ADAM9 gene and protein expression (*P*<0.05) (Figure 2D–F). Conversely, a marked increase in ADAM9 expression was observed in the miR-126a-3p inhibitor group compared with the negative control group (*P*<0.05). Such results proved that miR-126a-3p negatively regulates the expression of ADAM9.

### Arterial blood pressure and urine protein are significantly increased in pre-eclampsia

No significant difference was observed in the systolic blood pressure, diastolic pressure and urine protein of rats in the normal group and l-NAME group prior to treatment (all *P*>0.05). After treatment (18th day of gestation), the systolic blood pressure (108.95 ± 9.22 mmHg), diastolic pressure (80.17 ± 8.25 mmHg) and urine protein (6.59 ± 0.88 mg) of rats in the l-NAME group were up-regulated compared with the normal group (145.79 ± 15.24 mmHg, 105.33 ± 9.59 mmHg and 11.55 ± 1.28 mg, respectively) (all *P*<0.05), indicating that models were successfully constructed when pre-eclampsia-like signs appeared (Table 2).

**Table 2:** Comparison of blood pressure and urine protein levels in the two groups

	Treatment	*n*	Systolic pressure (mmHg)	Diastolic pressure (mmHg)	24-h urine protein (mg)
Control	Untreated	15	106.23 ± 8.94	80.15 ± 7.83	6.48 ± 0.79
	Normal saline injection	15	108.95 ± 9.22	81.17 ± 8.25	6.59 ± 0.88
l-NAME	Untreated	15	108.38 ± 10.25	81.04 ± 8.21	6.53 ± 0.74
	l-NAME injection	15	145.79 ± 15.24^1,2^	105.33 ± 9.59^1,2^	11.55 ± 1.28^1,2^
t_1_			8.672	7.877	13.05
P_1_			<0.05	<0.05	<0.05
t_2_			7.889	7.452	13.15
P_2_			<0.05	<0.05	<0.05

Blood pressure and urinary protein levels of each group were measured before and after model construction (at 6th and 18th days of gestation, respectively). *t* test was applied. ^1^Indicates *P_1_*<0.05 vs. Untreated. ^2^Indicates *P_2_*<0.05 vs. Control after treatment.

The article "miR-126a-3p induces proliferation, migration and invasion of trophoblast cells in pre-eclampsia-like rats by inhibiting A Disintegrin and Metalloprotease 9" was retracted in 2020. Reason: duplicated images.

### miR-126a-3p is down-regulated in the pre-eclampsia placenta

RNA *in situ* hybridization was performed to semi-quantify miR-126a-3p expression placental tissue from pre-eclampsia rats in the present study. The results suggested that miR-126a-3p is observed in the cytoplasm of trophoblast cells, vascular endothelial cells and smooth muscle cells of placental villi, which was significantly down-regulated in rats with pre-eclampsia (+) compared with normal rats (+++) (Figure 3).

**Figure 3:** RNA *in situ* hybridization of placental tissue Sample numbers of rats: pre-eclampsia, *n*=30; normal, *n*=10. The experiment was repeated three times.

### Identification of the isolation of placental trophoblast cells

Green fluorescence in the cytoplasm represents positive cells of cytokeratin 7 and vimentin, the blue fluorescence represents the DAPI-labeled nucleus. The results obtained from the immunofluorescence assay indicated that the majority of cells were positive to cytokeratin 7 at a percentage of 93.7%, while the percentage of vimentin-positive cells was 8.6%, confirming that cells obtained by separation and purification were the placental trophoblast cells of rats (Figure 4A,B).

**Figure 4:** Immunofluorescence staining of rat placental trophoblast cells (**A**) Immunofluorescence profile of Alexa Fluor® 488-labeled cytokeratin 7 and vimentin expression in trophoblast cells. (**B**) Percentage of cytokeratin 7 and vimentin-positive cells.

### miR-126a-3p down-regulates the expression of ADAM9 but increases cyclin D1, MMP-2 and MMP-9 content in trophoblast cells with pre-eclampsia

RT-qPCR and western blotting were applied to detect miR-126a-3p, mRNA and protein expression of ADAM9, cyclin D1, MMP-2 and MMP-9 in placental trophoblast cells in each group. The miR-126a-3p and ADAM9 expression indicated that miR-126a-3p regulates ADAM9 expression in its upstream pathway (miR-126a-3p is not affected by ADAM9 expression) (Figure 5A–C). Meanwhile, compared with the normal group, expression levels of cyclin D1, MMP-2 and MMP-9 were significantly decreased in all other groups (all *P*<0.05). Compared with the blank group, the miR-126a-3p mimic, siRNA-ADAM9 and miR-126a-3p mimic+siRNA-ADAM9 groups demonstrated a significant decrease in expression levels of cyclin D1, MMP-2 and MMP-9 (all *P*<0.05). Compared with trophoblast cells transfected with miR-126a-3p mimic or siRNA-ADAM9 separately, the aforementioned genes in the miR-126a-3p mimic+siRNA-ADAM9 group changed more significantly (all *P*<0.05). Compared with the blank group, the miR-126a-3p inhibitor group demonstrated a significant decrease in the levels of cyclin D1, MMP-2 and MMP-9 (all *P*<0.05). No significant differences in all genes were observed between the blank group and negative control group (all *P*>0.05) (Figure 5B,D,E). The aforementioned results indicated that stimulation of miR-126a-3p mimic could substantially decrease the content of ADAM9, but increase cyclin D1, MMP-2 and MMP-9 content in trophoblast cells with pre-eclampsia.

The article "miR-126a-3p induces proliferation, migration and invasion of trophoblast cells in pre-eclampsia-like rats by inhibiting A Disintegrin and Metalloprotease 9" was retracted in 2020. Reason: duplicated images.

**Figure 5:** Analysis reveals that stimulation of miR-126a-3p decreases ADAM9 but increases cyclin D1, MMP-2 and MMP-9 content in trophoblast cells with pre-eclampsia (**A,D**) Relative mRNA expression of miR-126a-3p, ADAM9, cyclin D1, MMP-2 and MMP-9 were determined by RT-qPCR. (**B**) Protein bands of ADAM9, cyclin D1, MMP-2 and MMP-9 in the trophoblast cells of each group following transfection. (**C**,**E**) The relative protein expression of ADAM9, cyclin D1, MMP-2 and MMP-9 was determined via Western blotting. ^∧^*P*<0.05 vs. Normal group; ^#^*P*<0.05 vs. negative control group; ^&^*P*<0.05 vs. miR-126a-3p mimic+siRNA-ADAM9 group. Sample numbers: Normal group, *n*=10; blank group, *n*=5; negative control, *n*=5; miR-126a-3p mimic group, *n*=5; miR-126a-3p inhibitor group, *n*=5; siRNA-ADAM9 group, *n*=5; and miR-126a-3p mimic+siRNA-ADAM9 group, *n*=5. The experiment was repeated three times.

### Stimulation of miR-126a-3p or ADAM9 knockdown results in effective promotion of placental trophoblast cell viability

The results of the MTT assay revealed that no significant difference was observed among all the groups at the 24th hour (all *P*>0.05). At the 48th and 72nd h, compared with the normal group, the other six groups exhibited decreasing trophoblastic cells viability (all *P*<0.05). Compared with the blank group, overexpressed miR-126a-3p or silencing of ADAM9 induced the proliferation of placental trophoblast cells in pre-eclampsia-like rats in a time-dependent manner, whereby, the effects were enhanced with the increase in time, and peaked at 72 h. The cell viability in miR-126a-3p mimic+siRNA-ADAM9 group increased more markedly when compared with the miR-126a-3p mimic and siRNA-ADAM9 groups (all *P*<0.05). No significant difference between the blank group and negative control group was observed (all *P*>0.05) (Figure 6). The results revealed that stimulation of miR-126a-3p mimic can inhibit the expression of ADAM9 and subsequently promote the viability of placental trophoblast cells in pre-eclampsia-like rats.

The article "miR-126a-3p induces proliferation, migration and invasion of trophoblast cells in pre-eclampsia-like rats by inhibiting A Disintegrin and Metalloprotease 9" was retracted in 2020. Reason: duplicated images.

**Figure 6:** Results of MTT assay indicate that the up-regulation of miR-126a-3p and ADAM9 silencing induces viability of trophoblast cells After transfection for 48 h, the trophoblast cells were seeded into 96-well plates and MTT assay was applied in order to detect the cell viability in each group. ^∧^*P*<0.05 vs. Normal group; ^#^*P*<0.05 vs. negative control group; ^&^*P*<0.05 vs. miR-126a-3p mimic+siRNA-ADAM9 group. Sample numbers: Normal group, *n*=10; blank group, *n*=5; negative control, *n*=5; miR-126a-3p mimic group, *n*=5; miR-126a-3p inhibitor group, *n*=5; siRNA-ADAM9 group, *n*=5; and miR-126a-3p mimic+siRNA-ADAM9 group, *n*=5. The experiment was repeated three times.

### Stimulation of miR-126a-3p or ADAM9 silencing relieves G_0_/G_1_ cell cycle arrest and induces the increase in S-phase cells

PI staining indicated that compared with the normal group, G_0_/G_1_ phase cells in other groups were increased, while cells in the S phase were decreased (all *P*<0.05). Compared with the blank group, G_0_/G_1_ phase cells were significantly decreased, while the S phase cells were increased in the miR-126a-3p mimic group, siRNA-ADAM9 group and miR-126a-3p mimic+siRNA-ADAM9 group (all *P*<0.05). Compared with the blank group, G_0_/G_1_ phase cells were significantly increased while S phase cells were decreased in the miR-126a-3p inhibitor group (all *P*<0.05). No significant difference was observed between the blank and negative control groups (all *P*>0.05). The miR-126a-3p mimic+siRNA-ADAM9 group exhibited a lower proportion of G_0_/G_1_ phase cells and a higher proportion of S phase cells compared with the miR-126a-3p mimic group and siRNA-ADAM9 group (all *P*<0.05) (Figure 7A,B). The results obtained from the cell cycle detection indicated that, miR-126a-3p stimulation or ADAM9 gene silencing could relieve the blockage of G_0_/G_1_ phase cells.

**Figure 7:** Up-regulation of miR-126a-3p and ADAM9 silencing relieves G_0_/G_1_ cell cycle arrest (**A**) Distribution of cell cycle in each group after transfection. (**B**) Histogram describing the cell cycle in each group. ^∧^*P*<0.05 vs. Normal group; ^#^*P*<0.05 vs. negative control group; ^&^*P*<0.05 vs. miR-126a-3p mimic+siRNA-ADAM9 group. Sample numbers: Normal group, *n*=10; blank group, *n*=5; negative control, *n*=5; miR-126a-3p mimic group, *n*=5; miR-126a-3p inhibitor group, *n*=5; siRNA-ADAM9 group, *n*=5; and miR-126a-3p mimic+siRNA-ADAM9 group, *n*=5. The experiment was repeated three times.

The article "miR-126a-3p induces proliferation, migration and invasion of trophoblast cells in pre-eclampsia-like rats by inhibiting A Disintegrin and Metalloprotease 9" was retracted in 2020. Reason: duplicated images.

### Stimulation of miR-126a-3p or ADAM9 silencing inhibits the apoptosis of placental trophoblast cells in pre-eclampsia-like rats

The cell apoptosis detection results revealed that, compared with the normal group, apoptosis in other groups was significantly up-regulated (all *P*<0.05). Compared with the blank group, cell apoptosis in the miR-126a-3p mimic group, siRNA-ADAM9 group and miR-126a-3p mimic+siRNA-ADAM9 group was significantly down-regulated, while cell apoptosis in the miR-126a-3p inhibitor group was increased (all *P*<0.05). No significant differences in cell apoptosis were observed between the blank and negative control groups (*P*>0.05). Cell apoptosis in the miR-126a-3p mimic + siRNA-ADAM9 group was decreased compared with the miR-126a-3p mimic group and siRNA-ADAM9 group (all *P*<0.05) (Figure 8A,B). Based on the aforementioned results, it can be concluded that miR-126a-3p or ADAM9 gene silencing could inhibit cell apoptosis of placental trophoblast cells in pre-eclampsia rats.

**Figure 8:** Up-regulation of miR-126a-3p and ADAM9 silencing inhibits the apoptosis of placental trophoblast cells (**A**) Scatter diagram showing the cell apoptosis in each group. (**B**) Percentage of apoptotic cells in each group. ^∧^*P*<0.05 vs. Normal group; ^#^*P*<0.05 vs. negative control group ^&^*P*<0.05 vs. miR-126a-3p mimic+siRNA-ADAM9 group. Sample numbers: Normal group, *n*=10; blank group, *n*=5; negative control, *n*=5; miR-126a-3p mimic group, *n*=5; miR-126a-3p inhibitor group, *n*=5; siRNA-ADAM9 group, *n*=5; and miR-126a-3p mimic+siRNA-ADAM9 group, *n*=5. The experiment was repeated three times.

### miR-126a-3p elevation combined with ADAM9 knockdown exhibits the most effective promotion of placental trophoblast cell migration

Wound healing assays were performed in order to determine the migration ability of trophoblast cells in each group. The results revealed that compared with the normal group, the other six groups demonstrated a marked decrease in the migration ability of trophoblast cells (all *P*<0.05). Compared with the blank group, the miR-126a-3p mimic, siRNA-ADAM9 and miR-126a-3p mimic+siRNA-ADAM9 groups demonstrated a significant elevation in the migration ability of trophoblast cells, and the miR-126a-3p mimic+siRNA-ADAM9 group exhibited the most effective increase in placental trophoblast cell migration (all *P*<0.05). No significant difference was observed in the negative control group when compared with the blank group (*P*>0.05) (Figure 9A,B).

The article "miR-126a-3p induces proliferation, migration and invasion of trophoblast cells in pre-eclampsia-like rats by inhibiting A Disintegrin and Metalloprotease 9" was retracted in 2020. Reason: duplicated images.

**Figure 9:** Wound-healing assay results revealed that stimulation of miR-126a-3p induces migration of trophoblast cells in rats with pre-eclampsia (**A**) Migration of trophoblast cells in each group after transfection for 48 h. (**B**) Percentage of migrated cells in each group. ^∧^*P*<0.05 vs. Normal group; ^#^*P*<0.05 vs. negative control group; ^&^*P*<0.05 vs. miR-126a-3p mimic+siRNA-ADAM9 group. Sample numbers: Normal group, *n*=10; blank group, *n*=5; negative control, *n*=5; miR-126a-3p mimic group, *n*=5; miR-126a-3p inhibitor group, *n*=5; siRNA-ADAM9 group, *n*=5; and miR-126a-3p mimic+siRNA-ADAM9 group, *n*=5. The experiment was repeated three times.

### miR-126a-3p elevation combined with ADAM9 knockdown exhibits the most effective promotion of placental trophoblast cell invasion

The transwell assay was utilized to analyze the invasive ability of trophoblast cells in each group. The results indicated that compared with the normal group, the other six groups showed a significantly decreased invasive ability (all *P*<0.05). Compared with the blank group, the miR-126a-3p mimic, siRNA-ADAM9 and miR-126a-3p mimic+siRNA-ADAM9 groups demonstrated an increased invasive ability, and the miR-126a-3p mimic+siRNA-ADAM9 group exhibited the most significant invasion ability (all *P*<0.05). However, no significant difference was detected between the blank and negative control groups (*P*>0.05) (Figure 10A,B). The aforementioned results indicate that stimulation of miR-126a-3p mimic or silencing of ADAM9 gene expression could enhance the migration and invasion of trophoblast cells in pre-eclampsia-like rats *in vitro*.

**Figure 10:** Transwell assay results suggest that stimulation of miR-126a-3p induces invasion of trophoblast cells in rats with pre-eclampsia (**A**) Migration of trophoblast cells in each group after transfection for 48 h. (**B**) Percentage of invasive cells in each group. ^∧^*P*<0.05 vs. Normal group; ^#^*P*<0.05 vs. negative control group; ^&^*P*<0.05 vs. miR-126a-3p mimic+siRNA-ADAM9 group. Sample numbers: Normal group, *n*=10; blank group, *n*=5; negative control, *n*=5; miR-126a-3p mimic group, *n*=5; miR-126a-3p inhibitor group, *n*=5; siRNA-ADAM9 group, *n*=5; and miR-126a-3p mimic+siRNA-ADAM9 group, *n*=5. The experiment was repeated three times.

## Discussion

Pre-eclampsia is a pregnancy-specific disorder, which markedly increases the chances of maternal mortality and mortality associated with pregnancy [26]. Despite previous investigations into pre-eclampsia, it remains to be a disease that cannot be completely cured. As the role of miRNAs continues to be elucidated, concerns are amounting with regard to miRNAs as a therapeutic option in pre-eclampsia. A previous study demonstrated that miR-137 could significantly decrease the migration and proliferation of trophoblast cells of pre-eclampsia, and it can serve as a potential target for gene therapy [23]. Another study revealed that abnormal expression of miR-210 may affect the function of trophoblasts, and miR-210 could be a promising therapeutic target for future pre-eclampsia treatment. These findings all supported the significance of miRNA therapeutics in pre-eclampsia [27]. The dysfunction of trophoblast cells is considered to be an important cause of pre-eclampsia [28]. Thus, the present study carefully designed a series of experiments to investigate the regulatory role of miR-126a-3p in placental trophoblast cells with the involvement of ADAM9. The results of the present study verified that miR-126a-3p can enhance the proliferation, migration and invasion ability of trophoblast cells by inhibiting the expression of ADAM9.

The article "miR-126a-3p induces proliferation, migration and invasion of trophoblast cells in pre-eclampsia-like rats by inhibiting A Disintegrin and Metalloprotease 9" was retracted in 2020. Reason: duplicated images.

Initially, the results of the bioinformatics analysis revealed that there was a differential expression of miR-126 in pre-eclampsia compared with the controls. A previous study indicated that miR-126 could be an efficient form of gene therapy to induce blood flow perfusion and blood vessel regeneration in pre-eclampsia [25]. As a result of the further analysis with the bioinformatics tools, ADAM9 was determined as the target gene that interacted with miR-126a-3p, and the present study aimed to reveal the molecular mechanism in which miR-126a-3p is involved in the pathogenesis of pre-eclampsia.

The results of the present study revealed that, compared with the Normal group, the expression of miR-126a-3p was significantly decreased in the placental trophoblast cells in the Model group. As an idiopathic hypertension syndrome, abnormal angiogenesis in the placenta is considered to be an important cause of pre-eclampsia. For this reason, pre-eclampsia is also considered to be a specific vascular complication during gestation [29]. A previous study highlighted that miR-126 is closely associated with lymphangiogenesis and angiogenesis in oral cancer [30]. Another study by Pitzler et al. [31] confirmed that miR-126a-3p could modulate the integrity of blood vessels by inducing ERK1/2 phosphorylation, thus stimulating the formation of perivascular cells. Another study concluded that overexpressed miR-126 could up-regulate the expression of VEGF in placental chorionic membrane cells with pre-eclampsia, which indicated that miR-126 may be involved in the morbidity of pre-eclampsia [32]. All these results suggest that down-regulation of miR-126 may be an important marker and potential therapeutic target in pre-eclampsia.

The article "miR-126a-3p induces proliferation, migration and invasion of trophoblast cells in pre-eclampsia-like rats by inhibiting A Disintegrin and Metalloprotease 9" was retracted in 2020. Reason: duplicated images.

Furthermore, in a study of pre-eclampsia and ADAM10, Hu et al. [33] revealed that the expression of ADAM10 in the placenta of patients with pre-eclampsia was significantly increased, which potentially resulted from the decrease in hydrogen sulfide (H_2_S) in the placenta. ADAM19 had also been reported to play an important role in the invasion of trophoblast cells [34]. In addition, a study that focused on the associations between ADAM10 and ADAM17 and pre-eclampsia trophoblast cells also confirmed that the Notch-2 intracellular domain of ADAM10 and ADAM17 could inhibit the migration and invasion of trophoblast cells [35]. The results obtained from the study by Ahmed et al. [16] revealed that 89.47% of pureperae with pre-eclampsia are subjected to ADAM9 gene mutations, suggesting that ADAM9 may be involved in the pathogenesis of pre-eclampsia.

In addition, the results of the luciferase assay, RNA pull-down and other experiments further confirmed that the involvement of ADAM9 in pre-eclampsia is associated with the regulation of upstream miR-126a-3p. Stimulation of miR-126a-3p mimic expression or silencing of ADAM9 gene expression can significantly promote the proliferation, migration and invasion of placental trophoblast cells in pre-eclampsia rats. Cyclin D1 is a well-recognized proto-oncogene that encodes cyclins and plays a positive regulatory role in cell proliferation [36]. It was revealed in a previous study that inhibition of cyclin D1 expression lead to insufficient cytotrophoblast invasion into the spiral artery, and then decreased cell invasion into decidua, leading to the formation of pre-eclampsia [37]. It can be speculated that the decreased expression of cyclin D1 in trophoblast cells in the Model group may be associated with the pathogenesis of pre-eclampsia. MMPs are proved to be involved in extracellular matrix remodeling and could degrade ECM through the function of protease, which in turn affects placental vascular remodeling and trophoblast cell invasion [38]. MMP-2 and MMP-9 are gelatinase proteins in the MMPs family. Deng et al. [39] confirmed that MGAT5 gene silencing promotes trophoblast cell invasion, which is closely associated with increased MMP-2/9 activity. Likewise, the present study observed that, compared with the Normal group, the expression of MMP-2 and MMP-9 in the placental trophoblast cells in the Model group was significantly decreased, which further confirmed that MMP-2 and MMP-9 plays a part in the pathogenesis of pre-eclampsia by participating in the proliferation of trophoblast cells. The flow cytometry assay further verified that miR-126a-3p stimulation or ADAM9 gene silencing could relieve the blockage of G_0_/G_1_ phase cells and inhibit the apoptosis of placental trophoblast cells. Therefore, the present study concluded that stimulation of miR-126a-3p mimic and silencing of ADAM9 could promote the proliferation, migration and invasion of trophoblast cells, but inhibit the apoptosis rate in rats with pre-eclampsia.

The article "miR-126a-3p induces proliferation, migration and invasion of trophoblast cells in pre-eclampsia-like rats by inhibiting A Disintegrin and Metalloprotease 9" was retracted in 2020. Reason: duplicated images.

In conclusion, the results of the present study provide a rationale for the hypothesis that miR-126a-3p could promote proliferation, migration and invasion, while inhibiting the apoptosis of trophoblast cells in pre-eclampsia-like rats through down-regulation of ADAM9 expression. miR-126a-3p is likely to be a potential therapeutic target against pre-eclampsia. However, the present study is still in the preclinical phase and so further investigation regarding the underlying molecular mechanism is still required in order to provide more reliable direction for future studies.

## Conclusion

In summary, results obtained from the present study demonstrated that miR-126a-3p could promote the proliferation, migration and invasion of trophoblast cells as well as inhibit trophoblast cells apoptosis through inhibiting ADAM9 in pre-eclampsia-like rats. miR-126a-3p is likely to be a potential therapeutic target against pre-eclampsia. The molecular mechanism of the present study is shown in Figure 11.

**Figure 11:** Molecular mechanism of miR-126-3p promotes the proliferation, migration and invasion of placental trophoblastic cells in pre-eclampsia rats through inhibiting ADAM9

## Ethic statements

The ethics approval (approval number: 2018-KY054-01) was obtained from the Animal Care and Use Committees of Beijing Obstetrics and Gynecology Hospital, Capital Medical University. Furthermore, total experimental operations on animals have been completed at above-mentioned hospital following the International Convention on Laboratory Animal Ethics and were performed in strict accordance with the Guide for the Care and Use of Laboratory Animals.

## Abbreviations

ADAM9: A Disintegrin and Metalloprotease 9
Ago2: Argonaute 2
CHAPS: 3-[(3-cholamidopropyl)-dimethylammonio]-1-propane-sulfonate
DAB: diaminobenzidine
DAPI: 4,6-diamino-2-phenyl indole
ECM: extracellular matrix
EP: Eppendorf
GAPDH: glyceraldehyde-3-phosphate dehydrogenase
HRP: horseradish peroxidase
L-NAME: L-nitro-arginine methylester
MMP: matrix metalloproteinase
MTT: 3-(4,5-Dimethylthiazol-2-yl)-2,5-diphenyltetrazolium bromide
NC: negative control
PI: propidium iodide
RT-qPCR: reverse transcription-quantitative PCR
SD: standard deviation
siRNA: small interfering RNA
TBST: tris-buffered saline and tween
3′UTR: 3′ untranslated region
